# Tooth Wear and Tribological Investigations in Dentistry

**DOI:** 10.1155/2022/2861197

**Published:** 2022-06-09

**Authors:** Ran Wang, Yuanjing Zhu, Chengxin Chen, Yu Han, Hongbo Zhou

**Affiliations:** Xiangya Stomatological Hospital & Xiangya School of Stomatology, Central South University, Changsha, 410008 Hunan, China

## Abstract

Dental or tooth wear is a physiological process in the life cycle of teeth. Loss of the occlusal surface may cause excessive tooth wear. Several factors may contribute to tooth wear with different intensities and duration in the oral cavity. The oral cavity is generally compared to a tribological system to determine the various types of wear between teeth and restorative materials and assess the amount of dental wear. However, it is challenging to investigate in vitro and in vivo wear owing to the complexity of tooth wear; thus, a clear correlation between in vitro and in vivo data could not be established. This review is aimed at providing an insight into the etiology of tooth wear and tribological investigations in dentistry.

## 1. Introduction

The loss of hard tooth tissue is defined as tooth wear, which depends on several complex mechanisms of wear, often obscuring its origin. Therefore, this notion is often unclear [1]. Physiological tooth wear does not generally cause subjective symptoms. With the progression of tooth wear, severe pathological signs and symptoms may occur [2]. Based on the differences in intensity, tooth wear describes all types of noncarious loss of tooth substance, such as abrasion, attrition, erosion, and abfraction. Abrasion is generated during contact between the teeth and other substances, while attrition is produced by tooth-to-tooth interaction. Moreover, erosion affects the tooth surface negatively owing to a chemical process. Abfraction occurs due to abnormal mechanical and chemical occlusal loading at the cervical enamel [3]. Thus, tooth wear is a complex, multifactorial phenomenon.

Since dentists have the greatest control over the selection of materials, many studies focused on improving the wear properties of dental biomaterials and protecting teeth from excessive wear. With the development of biomaterials, the study of dental tribology has been paid much attention [4]. Numerous wear simulation devices have been developed. The oral cavity is generally compared to a tribological system. The system consists of four elements [5]:

1. A solid body (a tooth)
2. The counterbody, usually a solid (for example, an object or an opposite tooth)
3. The part between the first and second elements called the interface element, which is usually a solid (e.g., food pellet particles) and a liquid (saliva) that acts as a lubricant
4. Air

Biomaterials are important for dental restorations. Metals, alloys, composites, and ceramics are widely used, but these materials have various problems compared to human tooth enamel. Therefore, to synthesize a material with properties similar to the human tooth enamel, it is necessary to have a deep understanding of tooth microstructure and its response to wear resistance of different biomaterials [6].

A full understanding of the process of tooth wear and the quantitative and qualitative assessment after tooth wear can help to comprehend the fundamental mechanisms underlying this process and elucidate the heterogeneity of biomaterials [7]. In this review, we provided an insight into tooth wear for scrutinizing wear investigations in dentistry, including the problems with these investigations.

## 2. Type of Tooth Wear

Tooth wear is increasing in the general population in recent decades, owing to the consumption of acidic beverages, enamel hypoplasia, and symptoms of increased stress, such as gastroesophageal reflux disease and bruxism [8]. Although many studies have investigated tooth wear, our understanding of its etiology and pathogenesis is still inadequate [9]. The four types of tooth wear are described below in detail.

By considering the underlying mechanisms of tooth wear, a tribological terminology for dental wear type has also been suggested (Table 1).

### 2.1. Attrition

Attrition is the mechanical damage to hard tissue due to the tooth-to-tooth contact [10], so it should, in principle, be defined as two-body abrasion. However, mechanistically, it cannot be differentiated from three-body abrasion, since enamel debris between the contacting surfaces during attrition can act as abrasive particles [11]. There are several principal theories regarding the etiology of attrition.

The principal theories are the following.

#### 2.1.1. Functional Theory

Kim et al. found that lateral movement (e.g., grinding movement) had significantly greater levels of tooth wear compared to vertical movement (e.g., chopping movement) [12].

#### 2.1.2. Bruxism

Bruxism is mainly regulated centrally and manifests as clenching or grinding and tooth surface loss [13, 14]. It is divided into three types: sleep bruxism, awake bruxism, and nonspecified bruxism [15]. Some medications and addictive substances that induce or aggravate bruxism are shown in Table 2. Bruxism is the most severe factor associated with commonly occurring tooth wear, as the force produced during bruxism is up to six times greater than that during normal mastication [16].

#### 2.1.3. Lack of Posterior Support

Missing posterior teeth can result in a horizontal deviation to the masticatory side with increased occlusal support, which is defined as masticatory predominance [17]. Sustained mastication predominance may cause abnormal tooth attrition, tooth fracture, and facial deformities [18, 19].

Besides dens evaginatus and developmental defects of enamel (DDE) caused by developmental anomalies, posterior crossbite and deep bite might increase the incidence and severity of dental attrition [20–22].

### 2.2. Abrasion

Dental abrasion is defined as the wear of teeth by any substance other than tooth substance, so it should, in principle, be defined as three-body abrasion [23]. In tribology, there are generally two types of abrasive wear with three bodies. The first type of abrasive wear occurs when two objects are far apart from each other so that the abrasive particles can move freely between surfaces like fluids. In contrast, the second type of abrasive wear occurs when the two objects are so close to each other that the abrasive particles are still trapped between the surfaces [24].

### 2.3. Abfraction

Abfraction, a new term coined by Grippo, is a type of noncarious cervical lesion (NCCL) [25]. It describes tooth tissue loss/damage along the gingival margin by flexure and failure of tooth tissue owing to excessive occlusal loads [26]. The lesions are not caused by a single factor but are the result of the comprehensive action of many factors [27]. They are typically wedge-shaped or V-shaped lesions, like abrasion lesions. Moreover, bacterial plaque accumulates on these lesions, causing tooth hypersensitivity and possibly affecting the pulp vitality [27]. However, cervical abfraction may extend subgingivally, thereby differentiating it from abrasion [28].

### 2.4. Erosion

Dental erosion is the chemical loss of mineralized tooth substances caused by exposure to acids not derived from oral bacteria [29]. The loss of surface tissue due to simultaneous and/or subsequent exposure to mechanical forces is known as erosive tooth wear (ETW) [29].

ETW can be due to extrinsic factors, intrinsic factors, or a combination of both. Extrinsic factors are usually related to dietary habits, unhealthy lifestyle, occupational hazards, or acid and other medications [30–33]. Intrinsic factors, including gastroesophageal reflux disease and eating disorders, are risk factors causing the chemical demineralization of the tooth tissues as a result of contact with the acidic contents of the stomach [34, 35].

## 3. Tribological Testing

Different dental materials were used in experimental analyses, and different authors developed various protocols for testing tooth wear using tribometers [24]. In 2001, the International Organization for Standardization (ISO) published a technical specification on wear test guidelines describing several methods for two- and/or three-body contact tests (Tables 3 and 4). The two-body wear device refers to the direct contact between the grinding material and the tested sample and simulates the oral chewing movement in a certain circular motion mode to reveal the properties and tooth wear mechanism of the material and the tooth [37]. Several two-body wear simulators have been designed and used to simulate tooth wear. The pin-on-disc tribometer is extensively used to perform two-body wear tests [38]. The three-body wear device adds food-simulating particles (artificial saliva, rice grains, grain shells, etc.) between the grinding materials to simulate chewing, to accurately reproduce the chewing environment [39].

Different two-body and three-body test methods differ in a few aspects, such as the load, the number of cycles, frequency of cycles, and abrasive medium (see Tables 3 and 4) [40]. The Alabama, ACTA, OHSU, Zurich, and MTS wear simulators have been used most frequently in studies. Some scholars found that the force exerted by the MTS wear simulator through the hydraulic actuator can be controlled and adjusted, and only the expensive MTS wear simulator is a qualified machine to test wear [7]. In contrast, the Willytec wear simulator not only can satisfy the requirements of GLP and FDA but also is an adequate and cost-effective tool to test wear [41].

## 4. Quantitative and Qualitative Evaluation

Quantitative assessment primarily depends on the depth and volume of wear at the occlusal contact areas, while qualitative assessment refers to the detailed topographic surface analysis. Therefore, several methods and macroscopic and microscopic techniques have been used to assess the loss/damage of the teeth and dental materials in vitro and in vivo. A comparison of all methods is shown in Table 5.

### 4.1. Three-Dimensional Optical Profilometer

Noncontact laser profilometry (NCLP) is the gold standard for detecting and quantifying the extent of surface wear in dental tribology [49–51]. Optical profilometry is an accurate and rapid technique that is used to provide qualitative and quantitative nanoscale data during repeated measurements of the same tooth area, irrespective of whether the surface is flat, curved, stepped, rough, or smooth [52, 53]. The device is used by a chromatic confocal sensor with a white light axial source for measuring with a scanning velocity of 2 m/s and a refraction index of 10,000. After each experiment, the measurement data were processed using the software for superimposition of scans and subtraction analysis, enabling absolute quantification of the surface [54] (Figure 1).

Yilmaz used a three-dimensional profilometer to evaluate the mean volume loss and depth of the surface of the specimen after tooth wear to investigate the two-body wear mechanism between teeth and dental materials [55]. The accurate quantification of the mean total volume of the wear surface is a prerequisite for informing the professional about the wear performance [56].

### 4.2. Surface Hardness and Nanoindentation Techniques

Surface hardness and nanoindentation techniques are the two commonly used methods for measuring the hardness of the tooth surface. Surface hardness or microindentation is a relatively mature and traditional method, whereas nanoindentation (also known as ultra-microindentation) is a new technique that is suitable to assess the extent of tooth wear [58]. Nanoindentation (NI) technology can be used to study the local mechanical properties under different loading states based on load-displacement data of indentations at a submicron scale [59]. The hardness and the elastic modulus of the enamel surface were measured using a diamond tip, and the indentation of each sample was performed in the continuous stiffness mode to investigate the dependence of the mechanical properties on depth and determine the hardening depth [60] (Figure 2).

Peng et al. used impact treatment and nanoindentation/scratch techniques to study the surface hardening b ehavior of tooth enamel under chewing load in vitro and to investigate its mechanism and antiwear effects [60]. Using this technique to measure mechanical properties at multiple locations of the same enamel sample is suitable because it can accurately measure mechanical properties of very small volumes, has a good spatial resolution, and is highly sensitive to changes that affect their values [61].

### 4.3. Microscopy Techniques

#### 4.3.1. Scanning Electron Microscopy (SEM)

Scanning electron microscopy (SEM) is ideal for studying the structure of tooth enamel because it can provide high-resolution images of hard surfaces [62]. SEM helps to analyze the sample surface by checking dimensional topography and distribution of exposed features due to the high-resolution power and large depth of focus of SEM; the image appears three-dimensional [63, 64] (Figure 3). Specimen preparation for SEM is complex. For analyzing samples with common scanning electron microscopes, moisture loss of specimens due to the necessary steps for preparing the specimens may lead to additional alterations of the eroded surface. To avoid the collapse of the fragile eroded enamel surface structure, freeze-drying of samples was suggested [65]. SEM investigations can be performed on both polished and unpolished native surfaces after gold sputtering. SEM can be coupled with energy-dispersive X-ray spectroscopy, which provides information about the composition of a specimen based on the characteristic X-rays emitted under electron bombardment. Energy-dispersive X-ray spectroscopy can be used to determine quantitative changes in elemental composition from eroded surfaces and cross-sections [66].

Levrini et al. conducted a study using SEM and analyzed several extracted human teeth. The study provided an overview of the distinctive morphological features and the microwear features of dental wear lesions, thus clarifying their clinical and diagnostic presentations and possible significance [67]. SEM is a powerful research tool, but since it requires high vacuum conditions and complex sample preparation, the application of SEM is limited. Environmental scanning electron microscopy is a better version of SEM. It can work in a gaseous environment and provides a new method for biological research [68].

#### 4.3.2. Confocal Laser Scanning Microscopy (CLSM)

CLSM is a nondestructive technique that can quantify and visualize erosive lesions [70]. The technology combines laser scanning with the capture of traditional visible light microscope images to produce a detailed 3D image of the surface [51] (Figure 4). Moreover, from the image, stack measurements of the differences in the height between the eroded and undamaged areas can be performed along with a qualitative assessment of the surface finish of the samples. Recent studies on early erosion wear have suggested that characterization of the enamel surface texture may be an appropriate target for therapeutic oral care products [71].

Austin et al. used CLSM to determine the optimal scale at which enamel surface textural changes from citric acid demineralization and salivary remineralization in vitro [72]. Faraoni et al. analyzed the morphology, surface roughness, and the step formed on the dental enamel using CLSM to study the effects of the stomach and duodenal fluid on dental enamel surfaces [73]. Early enamel erosion lesions can be effectively characterized by high-resolution optical surface measurement instrumentation and optimized surface texture analysis techniques [72]. With the development of microtechnology, CLSM is considered to be the most sensitive qualitative evaluation technique [74].

#### 4.3.3. Atomic Force Microscopy

As an important member of the scanning probe microscopy family, atomic force microscopy (AFM) has provided additional insights into the surface morphology of dental material and/or tooth surfaces [75]. The 3D data obtained from AFM measurements were evaluated visually and numerically [76]. This approach has many advantages; the most important is the ability to collect data for 3D surface analysis and phase type of data, as well as numeric data of surface properties or histogram analysis data [77] (Figure 5). Despite their complexities and irregularities, the three-dimensional morphology of biological structures can reveal fine anatomical details. The force curve reveals the relationship between the atomic force and the sample-tip distance; the slope of the force curve directly reflects the elasticity of the samples [78].

Mao et al. found differences between DGI-II and the normal dentin microstructure by AFM, which was used to indicate the wear behavior of DGI-II dentin [79]. Sample preparation for AFM is simpler than that for SEM. AFM can measure biological samples in the air, vacuum, or liquids at a high spatial resolution [80]. Therefore, the rough sample preparation technique does not damage the fragile samples [58]. The combination of atomic force microscopy and superresolution optics can provide simultaneous images with super time and spatial resolution in biological studies [78]. Due to improvements in its performance and function, AFM has played an important role in biological studies [78].

### 4.4. Quantitative Light-Induced Fluorescence (QLF)

Quantitative light-induced fluorescence (QLF) is a technique that is mainly used for the noninvasive detection of depth or progression of early caries [82–84]. In QLF, blue fluorescent light (405 nm; near-ultraviolet light) is reflected on the tooth surface using a long-pass filter (>520 nm) [85]. In QLF images, fluorescence is absent where minerals have been lost, for example, in dental hard tissues. Therefore, QLF can be used to quantify natural tooth wear by the difference in fluorescence intensity [85] (Figure 6).

Lee et al. found that enamel autofluorescence in QLF was related to the chemical composition of the enamel, particularly the inorganic-organic interface. Although the chemical composition of tooth enamel can only be detected in the laboratory, the fluorescence of tooth enamel detected by QLF can be evaluated in the dental clinic, and thus, it has implications in the field of tooth bleaching or esthetic restorative materials [86]. The rate of fluorescence loss measured using QLF is highly valuable for developing a nondestructive and longitudinal tool for in vitro, in situ, and in vivo applications [87].

### 4.5. Optical Coherence Tomography (OCT)

OCT is a noninvasive imaging method that uses light and eliminates the risk of radiation exposure [89]. Among the currently used methods, optical coherence tomography (OCT) has a significant advantage because it allows quantitative analysis of enamel thickness to be performed at the chairside [90] (Figure 7). Additionally, OCT can be used noninvasively to perform tomography scans and reconstruct enamel images in three dimensions without X-ray ionizing radiation [91–93].

Alghilan et al. found that CP-OCT and micro-CT demonstrated excellent comparability regarding enamel thickness measurements of the worn surfaces and verified that CP-OCT is a viable alternative for longitudinal evaluation of tooth wear in high-risk patients [90]. Notably, wear depth measurements using CP-OCT showed lower variability compared to micro-CT, which suggested that CP-OCT is better at estimating wear depth [90]. Scanning source OCT (SS-OCT) is the latest version of OCT, in which the light source is a tunable laser that scans light at near-infrared wavelengths for real-time imaging [89] (Figure 8). OCT can generate cross-sectional images of translucent or semitranslucent biological structures with microscopic level resolution. In dentistry, OCT imaging can be performed to effectively diagnose dental caries, NCCL, occlusal tooth wear, and other age-related changes in the tooth structure [89].

## 5. Conclusion

Tooth wear has multiple effects, involving the interaction of mechanical, chemical, and biological factors. As a clinical challenge, tooth wear should be identified rapidly and managed appropriately. Several devices and methods have been established to simulate the tooth wear environment; however, the process is extremely complex. Zhou and Jin suggested that future dental research should focus on the following aspects [4]:

1. More in vitro studies are needed to demonstrate the mechanisms of tooth wear, such as the correlations of tooth evolution, microstructure, dietary habit, dental tribological behavior, and the influence of complex salivary components
2. It is necessary to further investigate the application of oral wear resistance mechanisms in oral rehabilitation, such as new oral materials and oral care products, and improve wear resistance

Lanza et al. concluded that the keyword “tribology” or “biotribology” has limited use in dentistry; however, when used more extensively, it can benefit biotribology with the enhanced clarity in this area of research [5]. Therefore, the association between tribology and dentistry might become stronger in the future.

## Figures and Tables

**Figure 1:** High-resolution images were obtained at the nanometer scale by scanning across a changed pit in an enamel surface. The scale is in *μ*m [57].

**Figure 2:** Variations in the nanomechanical properties of the original, polished, and natural enamel surfaces with indentation depth: (a) hardness and (b) elastic modulus [60].

**Figure 3:** Human tooth assembly in the SEM holder [69].

**Figure 4:** The surface texture image analysis workflow based on the results of the area-scale analysis correlated with microhardness [72].

**Figure 5:** (a, b) Three-dimensional optical profilometer images; (c) an AFM image of molehills; (d) a 2D profile analysis of a molehill [81].

**Figure 6:** The quantitative light-induced fluorescence (QLF) image analysis process. (a) A representative fluorescence image of occlusal tooth wear. (b) A designed patch area around the wear. (c) A reconstructed image based on the fluorescence of the sound area. The blue line indicates the sound reference area, while the red line indicates the deactivated area. (d) The difference in the fluorescence between the original and reconstructed images. (e) The results of the analysis of the tooth wear area [88].

**Figure 7:** CP-OCT b-scan (left) and a-scan (right) analyses for measuring the enamel thickness [90].

**Figure 8:** Real-time cross-sectional imaging was performed for the anterior tooth using SS-OCT [89].

**Table 1:** A comparison of dental and tribological terminologies of tooth wear [24, 36].

Dentistry	Biotribology
Attrition	Delamination/fatigue wear
	Two-body abrasion
Abrasion	Three-body abrasion
	Adhesive wear
Erosion	Corrosive/chemical wear
Abfraction	Fatigue wear

**Table 2:** Medications and addictive substances [15].

Classes of medications	Phenethylamines
	Selective serotonin reuptake inhibitors
	Anticonvulsants
Addictive substances	Alcohol
	Heroin
	Methamphetamine
	Methylenedioxymethamphetamine
	Nicotine
	Piperazines

**Table 3:** Two-body wear methods and wear simulators.

Devices	Medium	Movement	Loading	Force	Frequency	Cycles
Zurich [42]	Water	Impact (+sliding)	Electromagnetic	49 N	1.7 Hz	120,000, 240,000, 640,000, and 1,200,000
BIOMAT [43]	Water	Impact (+sliding)	Cam+weight	20 MPa (225 N)	2 Hz	4,000
MTS [44]	Water	Sliding	Hydraulic	13.35 N	—	120,000, 240,000, 640,000, and 1,200,000
Willytec Munich and Muc3 [45]	Water or other	Gnashing, slippage, striking	Weight	50 N	Range (Hz)	120,000
Alabama localized [46]	PMMA beads	Impact+sliding	Spring	75.6 N	1.2 Hz	100,000, 200,000, 400,000
Pin-on-disc [24]	Water	Impact (+sliding)	Pin-on-disc machine	2-20 N	2 Hz	1-15,000

^∗^Based on [7].

**Table 4:** Three-body wear methods and wear simulators.

Devices	Medium	Movement	Loading	Force	Frequency	Cycles
ACTA [47]	Rice/millet seed shell suspension	Sliding	Spring	15 N	1.0 Hz	100,000–200,000
OHSU [48]	Poppy seeds/PMMA beads	Impact+sliding	Electromagnetic	Abrasion 20 N Attrition 70 N	1.2 Hz	50,000–100,000
Alabama generalized [46]	PMMA beads	Impact+sliding	Spring	75.6 N	1.2 Hz	100,000, 200,000, 400,000

^∗^Based on [7].

**Table 5:** A comparative analysis of macroscopic and microscopic techniques.

Techniques	Advantage	Limitation
3D optical profilometer [94, 95]	3D optical profilometer can show surface roughness and volume loss accurately and rapidly	3D optical profilometer could not detect and monitor the progression of tooth loss over time
Nanoindentation techniques [58, 96]	It is particularly useful when analyzing inhomogeneous surface as different regions of the surface can be identified and indented	The elastic modulus and hardness of teeth tissues are easily influenced by a large number of extrinsic variables, such as the method of preparing the specimen and its state of hydration
Scanning electron microscopy [66]	Scanning electron microscopy (SEM) can be combined with energy-dispersive X-ray spectroscopy (EDS) to measure quantitative changes in elemental composition on worn surfaces	Differences in the angulation of specimens in SEM influence such measurements
Confocal laser scanning microscopy [66, 71]	The advantages of CLSM are the high resolution (less than 300 nm in the *x* and *y* directions and 20 nm in the *z* direction) and fast recording of the surface topography	As with the other microscopy techniques, CSLM fails to record textural details
Atomic force microscope [66, 71]	It is suitable for measuring the early stage of enamel demineralization	It is very time-consuming
Quantitative light-induced fluorescence [58, 97]	The major strengths of the fluorescence techniques are that they are nondestructive (and therefore, surfaces can be monitored over time, in vivo or in vitro)	The exact mechanisms by which QLF measures erosion are unclear
Optical coherence tomography [66, 71]	It can therefore penetrate significantly deeper into samples than other subsurface techniques, providing an extremely high-quality 3D image that is nondestructive to the sample surface	In vivo accessibility and positioning of the probe are problematic
